# Prediction of Long-Term Survival Outcome by Lymph Node Ratio in Patients of Parotid Gland Cancer: A Retrospective study

**DOI:** 10.3389/fsurg.2022.903576

**Published:** 2022-05-11

**Authors:** Wen-Mei Jiang, Jian-Feng Xu, Jun Chen, Guo-Li Li, Yun-Fei Gao, Quan Zhang, Yan-Feng Chen

**Affiliations:** ^1^ Department of Head and Neck Surgery, Sun Yat-sen University Cancer Center, State Key Laboratory of Oncology in South China, Collaborative Innovation Center for Cancer Medicine, Guangzhou, Guangdong, China; ^2^ Department of Surgery, Dongguan Third Bureau Hospital, Dongguan City, Guangdong, China; ^3^ Department of Otolaryngology, The Seventh Affiliated Hospital of Sun Yat-sen University, Shenzhen, China

**Keywords:** Parotid gland cancer, lymph node ratio, survival, stage I–IV, SEER

## Abstract

**Background:**

Lymph node ratio (LNR) has been reported to reliably predict cancer-specific survival (CSS) in parotid gland cancer (PGC). Our study was designed to validate the significance of LNR in patients with PGC.

**Methods:**

Patients diagnosed with stage I–IV PGC were enrolled from Surveillance Epidemiology and End Results database (SEER, *N* = 3529), which is the training group, and Sun Yat-sen University Cancer Center database (SYSUCC, *N* = 99), the validation group. We used X-tile software to choose the optimal cutoff value of LNR; then, univariable and multivariable analyses were performed, assessing the association between LNR and CSS.

**Results:**

The optimal cutoff value of LNR was 0.32 by X-tile based on 3529 patients from SEER. Cox proportional hazard regression analysis revealed better CSS for patients with LNR ≤ 0.32 (adjusted hazard ratio [HR] 1.612, 95% confidence interval [95% CI] 1.286–2.019; *p* < 0.001) compared with patients with LNR > 0.32 in SEER. In the SYSUCC cohort, patients with LNR ≤ 0.32 also had better CSS over patients with LNR > 0.32 (*p* < 0.001). In N2 and N3 stage groups, patients with LNR ≤ 0.32 had superior CSS outcomes over those with the LNR > 0.32 group, but this benefit was absent in the N1 stage group.

**Conclusions:**

In conclusion, the lymph node ratio turned out to be an independent prognostic factor for cancer-specific survival of PGC in this study. This valuable information could help clinicians to evaluate the prognosis of PGC and suggest that adequate lymph node dissection is necessary.

## Introduction

Among head and neck cancers worldwide, salivary gland cancer has taken up 1%–5% (1). Also, parotid gland cancer (PGC) accounts for 70% of the whole salivary gland cancer, with 24 pathological subtypes (2–4). At present, surgery is the standard option for PGC, and adjuvant radiotherapy is suggested when indicated, which has been previously documented to improve the survival rate and local control effect (5–7). According to some published articles, the 5-year disease-free survival rate was 69%–93.6% (8, 9) and the 5-year overall survival (OS) rate was 76%–94.6% for PGC (9, 10). Nowadays, doctors evaluate treatment outcomes and assess patients’ survival by the standard of the TNM system (11). However, in the TNM system, the lymph node status alone might not reliably predict prognosis (12–14), and some previous studies have shown that the lymph node ratio (LNR, the number of positive lymph nodes divided by the number of neck lymph nodes dissected) is another prognostic factor for head and neck cancers (12, 14–16), even though the number of these studies are still few. According to these studies, patients with different LNR levels had various survival outcomes in the same pathological stage diseases. Practically, clinicians give suggestions on follow-up and the mode of adjuvant therapy based on the evaluation of patients’ survival outcomes.

Therefore, the necessity to precisely predict the prognosis of PGC patients is evident. Thus, we analyzed patients’ data obtained from Surveillance Epidemiology and End Results (SEER) and Sun Yat-sen University Cancer Center (SYSUCC) databases and intended to provide findings derived from different databases to verify the prognostic significance of LNR in PGC. In addition, this present study was designed to choose an appropriate value of LNR with improved prediction efficiency for long-term survival in PGC patients.

## Patients and Methods

### Patients

The study was approved by the Clinical Research Ethics Committee of Sun Yat-sen University Cancer Center (approval number: B2018-175-01), and the informed consent of patients was waived. A total number of 3529 patients who underwent parotidectomy between 2004 and 2015 were enrolled in this study retrospectively. Patients who were eligible for this cohort study were pathologically confirmed stage I–IV according to the 8th edition of the American Joint Committee on Cancer Staging Manual. In addition, these patients were included in this study who met the following conditions: (1) pathologically diagnosed with parotid gland cancer, (2) one primary only, (3) surgical resection was not performed; and (4) complete follow-up. The exclusion criteria are shown in Figure 1.

**Figure 1:** Diagram of the patient screening process in the Surveillance Epidemiology and End Results and our center databases.

Furthermore, the data derived from the SYSUCC database were used to validate the results from SEER. According to similar screening criteria, there were 99 patients selected from the SYSUCC database as an external validation cohort. These patients took operation between 1999 and 2016. The flow chart of the study is shown in Figure 1.

### Follow-up

In the SEER database, the median follow-up time was 45 months (range 0–155 months). At SYSUCC, those patients were followed up by telephone regularly by the professional follow-up department. The median follow-up time with patients from surgery to the last contact was 64 months (range 1–195 months). The last follow-up date was February 20, 2020, and no patients were lost to follow-up.

### Statistical analysis

Statistical analysis was performed using SPSS Statistics 25.0 software (IBM SPSS, Inc., Chicago, IL, USA) and X-tile version 3.6.1 (http://www.tissuearray.org/rimmlab). X-tile software was conducted to choose the optimal cutoff point of LNR (17). Previous studies have shown that X-tile software was similar to the time-varying receiver operating characteristic curve analysis and could provide the best cutoff value for continuous data (18, 19). Chi-squared tests and Fisher exact tests were applied to evaluate the association between clinical variables and LNR groups of different levels. Hazard ratios (HRs) with 95% confidence interval (CI) were calculated by univariable and multivariable Cox proportional hazard regression analyses. Univariable and multivariable analyses were performed to evaluate the effect of sex, age, LNR, marital status, grade, radiotherapy, chemotherapy, race, drinking history, pathological N (pN) stage, pathological T (pT) stage, smoking history, and histological subtypes on CSS. Variables with *p* < 0.05 in univariable analysis or affecting prognosis (such as sex, approaches of treatment, and tumor differentiation) were selected to enter the multivariable analysis to further confirm the independent prognostic factors. Additionally, Kaplan–Meier analysis and log-rank tests were applied to compare survival curves between groups. The point of CSS as a primary clinical endpoint was considered most clinically relevant, and it was statistically considered significant when the results of all statistical tests met a two-sided *p *< 0.05. Patients from the SYSUCC database were stratified using the cutoff point of LNR defined in the SEER data set into two subgroups.

## Results

### Patient Characteristics

The clinical characteristics of the patients from the SEER database are listed in Table 1. Among the 3529 cases, 2033 (57.6%) of them were men and 1496 (42.4%) of them were women (male vs. female = 1.36:1). The age ranged from 18 to 104 years (median, 60 years). In the SEER cohort, the 1-, 3-, and 5-year CSS rates were 92.0%, 87.0%, and 84.0%, respectively, with the median survival time of 44 months. Lymph node metastasis was reported in 1188 cases (33.7% of the SEER cohort). The optimal cutoff value of LNR was determined by X-tile as 0.32 based on the SEER database.

**Table 1:** Patient characteristics in Surveillance Epidemiology and End Results database.

Variables	LNR		*p*-value
	≤0.32 (*N* = 3063)	>0.32 (*N* = 466)	
**Sex**			<0.001*
Male	1716 (56.0%)	317 (68.0%)	
Female	1347 (44.0%)	149 (32.0%)	
**Age (years)**			<0.001*
≤65	1958 (63.9%)	231 (49.6%)	
>65	1105 (36.1%)	235 (50.4%)	
**Marital status**			0.647*
No	1140 (37.2%)	167 (35.8%)	
Yes	1778 (58.1%)	280 (60.1%)	
Unknown	145 (4.7%)	19 (4.1%)	
**pT stage**			<0.001**
T1	1032 (33.7%)	61(13.1%)	
T2	893 (29.2%)	100 (21.5%)	
T3	583 (19.0%)	143 (30.7%)	
T4	555 (18.1%)	162 (34.8%)	
**pN stage**			<0.001**
N0	2337 (76.3%)	0 (0.0%)	
N1	348 (11.4%)	156 (33.5%)	
N2	369 (12.0%)	301 (64.6%)	
N3	9 (0.3%)	9 (1.9%)	
**Pathological subtypes**			<0.001*
Adenoid cystic carcinoma	239 (7.8%)	19 (4.1%)	
Adenocarcinoma	980 (32.0%)	136 (29.2%)	
Mucoepidermoid carcinoma	824 (26.9%)	66(14.2%)	
Squamous cell carcinoma	525 (17.1%)	103 (22.1%)	
Myoepithelial carcinoma	120 (3.9%)	4 (0.9%)	
Ductal carcinoma	69 (2.3%)	46 (9.8%)	
Other subtypes	306 (10.0%)	92 (19.7%)	
**Radiotherapy**			<0.001*
No	1278 (41.7%)	99 (21.2%)	
Yes	1785 (58.3%)	367 (78.8%)	
**Chemotherapy**			<0.001*
No	2736 (89.3%)	300 (64.4%)	
Yes	327 (10.7%)	166 (35.6%)	
**Tumor grade**			<0.001*
Grade I	482 (15.7%)	10 (2.1%)	
Grade II	829 (27.1%)	54 (11.6%)	
Grade III	659 (21.5%)	228 (48.9%)	
Grade IV	323 (10.5%)	92 (19.7%)	
Unknown	770 (25.2%)	82 (17.7%)	
**Race/ethnicity**			0.132*
White patients	2472 (80.7%)	385 (82.6%)	
Black patients	293 (9.6%)	30 (6.4%)	
Other patients	272 (8.9%)	48 10.3%)	
Unknown	26 (0.8%)	3 (0.7%)	

*LNR, lymph node ratio.*

* Chi-squared test; **Fisher’s exact test.

In the SYSUCC cohort, the 1-, 3-, and 5-year CSS rates were 81.0% vs. 72.0% vs. 68.0%, respectively, and the median survival time was 63 months. The clinical characteristics of the SYSUCC cohort are listed in Table 2. Of the whole 99 patients, 43 cases (43.4% of the SYSUCC cohort) with pathologically positive lymph nodes.

**Table 2:** Patient characteristics in our center database.

Variables	LNR		*p*-value
	≤0.32 (*N* = 78)	>0.32 (*N* = 21)	
**Sex**			0.137*
Male	27 (34.6%)	11 (52.4%)	
Female	51 (65.4%)	10 (47.6%)	
**Age (year)**			0.064*
≤65	71 (91.0%)	16 (76.2%)	
>65	7 (9.0%)	5 (23.8%)	
**Smoking history**			0.040**
No	73 (94.8%)	17 (81.0%)	
Yes	4 (5.2%)	4 (19.0%)	
**Drinking history**			0.936**
No	73 (94.8%)	20 (95.2%)	
Yes	4 (5.2%)	1 (4.8%)	
pT stage			0.790**
T1	8 (10.3%)	1(4.8%)	
T2	16 (20.5%)	4 (19.0%)	
T3	14 (17.9%)	3 (14.3%)	
T4	40 (51.3%)	13 (61.9%)	
**pN stage**			<0.001**
N0	55 (70.5%)	0 (0.0%)	
N1	9 (11.5%)	4 (19.0%)	
N2–3	14 (18.0%)	17 (81.0%)	
**Type of resection**			0.005**
R0	76 (97.4%)	17 (81.0%)	
R1/R2	2 (2.6%)	4 (19.0%)	
**Radiotherapy**			0.314**
No	77 (98.7%)	20 (95.2%)	
Yes	1 (1.3%)	1 (4.8%)	
**Chemotherapy**			0.001**
No	76 (97.4%)	16 (76.2%)	
Yes	2 (2.6%)	5 (23.8%)	
**Pathological subtypes**			<0.001*
Adenoid cystic carcinoma	16 (20.5%)	0 (0.0%)	
Adenocarcinoma	17 (21.8%)	2 (9.5%)	
Mucoepidermoid carcinoma	18 (23.1%)	5 (23.8%)	
Squamous cell carcinoma	4 (5.1%)	5 (23.8%)	
Myoepithelial carcinoma	2 (2.6%)	0 (0.0%)	
Ductal carcinoma	1 (1.3%)	0 (0.0%)	
Other subtypes	20 (25.6%)	9 (42.9%)	
**Tumor grade**			0.124*
Grade I	6 (30.0%)	1 (11.1%)	
Grade II	8 (40.0%)	1 (11.1%)	
Grade III	5 (25.0%)	6 (66.7%)	
Grade IV	1 (5.0%)	1 (11.1%)	

*LNR, lymph node ratio.*

* Chi-squared test; **Fisher exact test.

### Univariable and Multivariable Analyses of SEER

As shown in Table 3, univariable and multivariable analyses identified the following variables as independent prognostic factors for PGC patients: LNR (adjusted HR 4.778, 95% CI 3.936–5.802; *p* < 0.001), sex, age, radiotherapy, chemotherapy, pT stage, pN stage, tumor grade, and pathological subtypes. Our results revealed that the 12-month, 36-month, and 60-month CSS rates in the subgroup of LNR > 0.32 were 75%, 61%, and 56% compared to 95%, 81%, and 88% in the subgroup of LNR ≤ 0.32. We found that there was a statistically significant difference in CSS rates between the LNR ≤ 0.32 and LNR > 0.32 group (Figure 2A, unadjusted HR 4.778, 95% CI, 3.936–5.802, log-rank test: *p* < 0.001).

**Figure 2:** Cancer-specific survival curves for parotid gland cancer patients according to the lymph node ratio in the cohort of Surveillance Epidemiology and End Results database (**A**) and our center database (**B**).

**Table 3:** Univariable and multivariable Cox proportional hazard regression analyses for overall survival in parotid gland cancer patients with stage I–IV from Surveillance Epidemiology and End Results database.

	Univariable analysis			Multivariable analysis		
	HR	95% CI	*p*-value	HR	95% CI	*p*-value
**Sex**						
Male vs. female	0.593	0.487–0.722	<0.001	0.942	0.765–1.161	<0.577
Age (years)						
≤65 vs. >65	2.256	1.872–2.717	<0.001	1.559	1.276–1.904	<0.001
**LNR**						
≤0.32 vs. >0.32	4.778		<0.001	1.612	1.286–2.019	<0.001
**Marital status**						
No	1	Reference				
Yes	1.138	0.934–1.387	0.199			
Unknown	0.738	0.427–1.276	0.277			
**pT stage**						
T1	1	Reference		1	Reference	
T2	2.899	2.002–4.197	<0.001	2.244	1.546–3.258	<0.001
T3	5.734	4.006–8.206	<0.001	2.745	1.895–3.978	<0.001
T4	10.151	7.221–14.272	<0.001	4.413	3.090–6.303	<0.001
**pN stage**						
N0	1	Reference				
N1	4.156	3.208–5.385	<0.001	2.022	1.516–2.698	<0.001
N2	7.806	6.268–9.723	<0.001	2.764	2.087–3.660	<0.001
N3	6.437	2.635–15.726	<0.001	1.890	0.757–4.714	0.172
**Pathological subtypes**						
Adenoid cystic carcinoma	1	Reference		1	Reference	
Adenocarcinoma	1.124	0.758–1.666	0.561	0.902	0.597–1.364	0.625
Mucoepidermoid carcinoma	0.701	0.458–1.072	0.101	0.661	0.420–1.042	0.074
Squamous cell carcinoma	1.763	1.171–2.656	0.007	0.720	0.459–1.129	0.153
Myoepithelial carcinoma	0.360	0.140–0.929	0.035	0.461	0.178–1.197	0.112
Ductal carcinoma	2.519	1.489–4.261	0.001	0.638	0.365–1.116	0.115
Other subtypes	2.028	1.327–3.101	0.001	0.759	0.480–1.201	0.239
**Radiotherapy**						
No vs. yes	2.540	2.014–3.203	<0.001	1.043	0.815–1.335	0.739
Chemotherapy						
No vs. yes	3.347	2.739–4.090	<0.001	1.313	1.046–1.647	0.019
**Tumor grade**						
Grade I	1	Reference		1	Reference	
Grade II	5.637	2.588–12.279	<0.001	3.449	1.575–7.554	0.002
Grade III	19.964	9.394–42.428	<0.001	5.365	2.473–11.641	<0.001
Grade IV	21.252	9.885–45.689	<0.001	6.416	2.930–14.049	<0.001
Unknown	5.886	2.709–12.789	<0.001	3.541	1.614–7.768	0.002
**Race/ethnicity**						
White patients	1	Reference		1	Reference	
Black patients	0.758	0.536–1.072	0.117	1.011	0.709–1.441	0.952
Other patients	0.627	0.435–0.904	0.012	0.765	0.525–1.114	0.162

*LNR, lymph node ratio; Cox regression’s method was Enter selection. The number of patients of unknown races was too few to perform analysis.*

### Validation for the Survival Impact of LNR in the SYSUCC Database

In order to validate the impact of LNR on CSS in parotid gland cancer patients, we enrolled another 99 patients from SYSUCC as an external cohort. We stratified the patients within this validation group into the subgroup of LNR > 0.32 and the subgroup of LNR ≤ 0.32, and the latter was found with worse CSS outcomes (unadjusted HR 2.657, 95% CI, 1.319–5.351, log-rank test: *p* = 0.00045, Figure 2B). Our results revealed that the 12-month, 36-month, and 60-month CSS rates in the subgroup of LNR > 0.32 were 54%, 48%, and 44% in the subgroup of LNR > 0.32 compared to 88%, 78%, and 74% in the subgroup of LNR ≤ 0.32.

### Subgroup Analysis for CSS

The N stage was an important factor in affecting survival (Table 3). After adjusting for other confounders, LNR was confirmed to be an independent prognostic factor in the present study (Table 3). Based on the results of multivariable Cox proportional hazard regression analyses, a nomogram for prognostic prediction was established for the SEER cohort (Figure 3). The visual nomogram showed the weights of variables affecting the prognosis of PGC.

**Figure 3:** Nomogram to show the weights of variables affecting survival.

To investigate the association between LNR and N stage, we performed the Kaplan–Meier method to compare the survival of patients with different LNR levels in the cohorts with stages N1, N2, and N3. The results showed that in N2 and N3 stage groups, patients with LNR ≤ 0.32 had superior CSS outcomes over those with the LNR > 0.32 group, but this benefit was absent in the N1 stage group (Figure 4). Besides, our results showed that LNR could be a risk indicator among the population of different histological subtypes except for the cohort with other subtypes (all *p*’s < 0.05, Figure 5). Limited by the number of patients, the subgroup survival curve was not drawn in our center. Our results showed that unadjusted HR exceeded 1 or, in other words, LNR > 0.32 could be a risk indicator among the population of different histological subtypes except for cohorts with other subtypes (Figure 5).

**Figure 4:** Cancer-specific survival curves for parotid gland cancer patients with stage N1 (**A**), N2 (**B**), and N3 (**C**) according to the lymph node ratio in the cohort of Surveillance Epidemiology and End Results database and Sun Yat-sen University Cancer Center.

**Figure 5:** Impact of lymph nodes ratio on survival in population with different characteristics.

## Discussion

In the present study, we analyzed the data of patients with PGC from two research databases: SYSUCC and SEER. The data of SEER was set as the training group and analyzed by univariable and multivariable Cox regression, and then, the results were validated in the SYSUCC database. LNR and tumor grading were considered independent prognostic factors, and in this study, we found that LNR ≤ 0.032 was associated with better CSS for patients with PGC. Furthermore, LNR was found to be a prognostic indicator among the population of different histological subtypes except for cohorts with other subtypes and LNR was also identified to have an excellent discriminated efficiency in stage III–IV groups and each T stage by the subgroup analysis. Actually, the relative data for LNR could be easily obtained from the medical record, which makes it rather practical to validate our results by multi-institution study and be applied in clinical work.

Previous studies had revealed that LNR could be a prognostic indicator for PGC patients. Meyer et al. retrospectively analyzed the medical data of 128 patients with PGC by multivariable Cox regression and suggested that LNR < 0.1 was an independent protective prognostic factor for OS (HR, 0.332, *p* = 0.043) (13). However, the TNM stage was not a significant prognostic factor in their study after adjusting for other factors. Another study by Elhusseiny et al. revealed that LNR > 0.3333 was a risk prognostic factor for major salivary gland cancer, including 4608 PGC patients (20). In addition, the diseases’ stage was also proved an independent prognosticator for this malignancy in Elhusseiny’s research. As for our study, T stage, N stage, and LNR were both proved to be independent prognostic factors by analyzing the SEER data. Our findings were similar to Elhusseiny’s, and different from Meyer’s, and his disparity might be derived from the difference in sample size. In Meyer’s study, adjuvant radiotherapy followed surgery did not provide a survival benefit for PGC patients. The findings were similar to our results. The results of the present study revealed that radiotherapy could not serve as a protective prognostic factor for PGC patients after adjusting for other confounders. Besides, Elhusseiny’s study did not conclude that adjuvant radiotherapy is a protective factor for PGC patients. Our research excluded patients who did not receive surgery and patients whose number of lymph-node-dissection areas was less than one. Elhusseiny’s research included patients without surgery yet and did not restrict the lymph-node-dissection area on patients. Though our patient screening process was different from theirs, we got similar findings. Therefore, prospective studies are still needed to demonstrate the significance of radiotherapy in patients undergoing surgical resection of PGCs.

We also found that histological subtypes could significantly affect the CSS by analyzing the data of the SEER database. However, the results in the univariable analysis and multivariable analysis were not exactly consistent. In the results of univariable analysis, squamous cell carcinoma, ductal carcinoma, and other subtypes were considered risk indicators affecting CSS, while myoepithelial carcinoma was associated with better CSS (Table 3). However, after adjusting for other confounders, the pathological subtypes did not play a role in impacting the survival of PGC patients. In fact, the mucoepidermoid carcinoma and myoepithelial carcinoma were seen as low-risk histological subtypes according to the risk stratification of WHO-recognized salivary gland malignancies, which were not prone to lymph node metastasis (21). Qian et al. suggested that histological subtypes could affect the cancer-specific survival of salivary gland cancer patients independently (22). However, in this study, we could not conclude similar conclusions to theirs. The first reason might be that the selected cases of the two studies were different. We selected patients with PGC; however, they selected patients with all salivary gland carcinoma. The second reason was that they classified pathological subtypes as high- and low-risk groups; however, we separated each subtype in order to explore the role of LNR in different pathological subtypes. Therefore, we suggest that future research should focus on the influence of pathological subtypes on the prognosis of PGC patients.

There are some limitations to our study. First, the sample size of PGC patients was relatively limited in the SYSUCC database, and the data distribution of the TNM stage was not balanced in the two databases. Therefore, the data of SYSUCC were only used to perform the Kaplan–Meier analysis in order to validate the results from the SEER database. To improve this aspect, the sample size would need to be expanded in further studies. Second, the patients’ data used in this study originated from limited academic databases, which might also impact the accuracy of our findings, so a larger scale of patients’ information from multiple centers was necessary to confirm our results. Third, these findings could only provide certain reference information to the clinicians but not the treatment recommendations. Doctors would need to make decisions on the patients’ treatment according to the relevant guidelines and clinical experience. Fourth, data on molecular diagnosis were absent, which might be effective prognostic factors contributing to a more accurate prediction. Therefore, substantial research at the molecular level is still needed to further improve the proposed findings.

## Conclusions

In conclusion, the lymph node ratio turned out to be an independent prognostic factor for cancer-specific survival in this study. This valuable information could help clinicians evaluate the prognosis of parotid gland cancer and suggest that adequate lymph node dissection is necessary.

## Data Availability

The raw data supporting the conclusions of this article will be made available by the authors without undue reservation.
